This article has been retracted.

# Proanthocyanidins Antagonize Arsenic-Induced Oxidative Damage and Promote Arsenic Methylation through Activation of the Nrf2 Signaling Pathway

**DOI:** 10.1155/2019/8549035

**Published:** 2019-01-20

**Authors:** Mengchuan Xu, Qiang Niu, Yunhua Hu, Gangling Feng, Haixia Wang, Shugang Li

**Affiliations:** Department of Public Health, Medical College, Shihezi University, 832000 Xinjiang, China

## Abstract

**Purpose:**

To investigate the effects of grape seed proanthocyanidin extract (GSPE) on oxidative damage and arsenic (As) methylation and to clarify the role of Nrf2 in the process.

**Methods:**

L-02 cells were treated with arsenic (25 *μ*M) and GSPE (10, 25, and 50 mg/L) for 24 h. Cell viability was analyzed by MTT assay. Cell apoptosis and ROS fluorescence were detected by flow cytometry. Oxidative stress marker levels were measured using commercial kits. mRNA and protein expression were detected by qRT-PCR and western blotting. The cellular concentrations of methylation products were measured by HPLC-HGAFS. Arsenic methylation ability of cells was determined.

**Results:**

Cell survival rate was significantly lower in the As group than in the control group (*P* < 0.05), while cell apoptosis increased and the number of apoptotic cells decreased gradually after GSPE intervention. Superoxide dismutase, glutathione, and sulfhydryl levels in the intervention group were significantly higher (*P* < 0.05), while MDA and ROS levels were significantly lower (*P* < 0.05) than those in the As group. The mRNA and protein expression of Nrf2, HO-1, NQO1, and glutathione-S-transferase increased in the As + GSPE group compared with that in the As group (*P* < 0.05). GSPE significantly increased methylated As level, primary methylation index, secondary methylation index, average growth rate of methylation, and average methylation speed compared with the GSPE untreated group (*P* < 0.05). After Nrf2 inhibition, the effect of GSPE decreased significantly.

**Conclusion:**

GSPE activates the Nrf2 signaling pathway to antagonize As-induced oxidative damage and to promote As methylation metabolism. Therefore, GSPE may be a potential agent for relieving As-induced hepatotoxicity.

## 1. Introduction

Arsenic is a metalloid toxin and carcinogen present widely in soil, rocks, and water [1]. Our previous studies have proved that arsenic can cause reproductive toxicity [2, 3], but the mechanism of arsenic toxicity is not completely clear and should be further studied. In recent years, China has gradually become one of the countries with the highest impact and incidence rate of endemic arsenism [4].

The liver is one of the important target organs of arsenic toxicity. Arsenic is mainly metabolized by methylation in the liver [5]; however, the methylation of arsenic is not exactly a detoxification process. Arsenic methylation is regulated by glutathione (GSH). The toxicity of monomethylarsonic acid (MMA)^3+^ produced by arsenic metabolism is much higher than that of inorganic arsenic (iAs). Different metabolism levels of arsenic methylation may be an important reason for arsenic-induced liver damage. Lipid peroxidation caused by oxidative stress is considered one of the important mechanisms of arsenic poisoning [6]. Therefore, antagonizing the toxicity of arsenic through antioxidation has become an important breakthrough in the prevention and control of arsenic poisoning. Nuclear factor E2-related factor (Nrf2), which is regulated by Kelch-like ECH-associated protein-1 (Keap1), is an important regulatory factor of cell resistance to oxidative stress [7]. Nrf2 can regulate various antioxidant enzymes, such as glutathione-S-transferase (GST), heme oxygenase 1 (HO-1), NADPH: quinone oxidoreductase-1 (NQO1), and *γ*-glutamate-cysteine ligase (*γ*-GCL) [8], to improve the antioxidant capacity of the body.

Proanthocyanidins can effectively remove various reactive oxygen species (ROS) and have many biological activities, such as antioxidant, free radical scavenging [9], antitumor, cardiovascular protective, and cell proliferative effects [10]. Up till now, there are many health products containing proanthocyanidins in the domestic and foreign markets, such as proanthocyanidin capsule and grape seed antioxidant [11]. Proanthocyanidins can be added to yogurt, cakes, and other foods as a food supplement. In addition, proanthocyanidins are widely used in cosmetics, such as hand cream and sunscreen cream [12].

Many animal experiment data [13–15] have shown that proanthocyanidins could decrease the content of malondialdehyde (MDA), increase the levels of antioxidant enzymes, such as glutathione peroxidase (GSH-PX), catalase (CAT), and superoxide dismutase (SOD), and alleviate the oxidative damage induced by zearalenone, aflatoxin B1, and lead in mice. Cell experiments [16, 17] and clinical trials [18, 19] have also shown that proanthocyanidins can effectively reduce oxidative product levels and increase the total antioxidant capacity (T-AOC). Proanthocyanidins, as a natural and efficient free radical scavenger and antioxidant, can help the body to resist lipid peroxidation induced by environmental factors. On the one hand, oxidative stress is an important reason for arsenic-induced liver injury. On the other hand, it can regulate cytotoxicity caused by arsenic methylation metabolism.

Grape seed proanthocyanidin extract (GSPE) has high antioxidant activity. However, it is not clear whether proanthocyanidins antagonize arsenic toxicity through the Nrf2 pathway in L-02 cells. In addition, the effects of proanthocyanidins on arsenic methylation metabolism have not yet been reported. In our study, L-02 cells were treated with arsenic and/or GSPE for 24 h. We evaluated the antagonistic effect of proanthocyanidins on liver cell toxicity induced by arsenic and explored the possible mechanism by which proanthocyanidins antagonized arsenic-induced oxidative damage of hepatocytes. The findings of this study provide a basis for the development and utilization of grape seed procyanidin resources and a reference for the prevention and control of endemic arsenic poisoning in Xinjiang.

## 2. Materials and Methods

### 2.1. Materials and Reagents

Standards of iAs^3+^ (NaAsO_2_), iAs^5+^, sodium methyl arsenate, and sodium dimethylarsinate were purchased from Sigma-Aldrich Co. (San Francisco, USA). Commercially available GSPE powder was obtained from Solarbio Science & Technology Co. Ltd. (Beijing, China; purity ≥ 95%). Human hepatocytes (L-02 cells) were purchased from Obio Technology Co. Ltd. (Shanghai, China).

SOD, GSH, MDA, sulfhydryl (-SH), alanine aminotransferase (ALT), aspartate aminotransferase (AST), and ROS kits were purchased from Nanjing Jiancheng Bioengineering Institute (Nanjing, China). Anti-Nrf2, anti-HO-1, anti-NQO1, and anti-GST antibodies were obtained from Abcam Ltd. (Abcam, Cambridge, UK). ML385 (Lot no. 846577-71-9), an Nrf2 inhibitor, was purchased from MedChemExpress (New Jersey, USA).

Dulbecco's modified Eagle's medium (DMEM), hyperglycemic medium, fetal bovine serum (FBS), and trypsin were all purchased from Gibco (California, USA).

### 2.2. Cell Culture

L-02 cells were cultured in DMEM containing 100 U/mL penicillin, 100 mg/mL streptomycin, and 10% (*v*/*v*) FBS. The cells were cultured in 25 cm^2^ flasks and seeded onto 6-well tissue culture plates at 37°C with 5% CO_2_. The medium was replaced every 2 days until the cells reached 80–90% confluence (3–5 days). After reaching 80–90% confluence, arsenic (final concentration 0 and 25 *μ*mol/L) and/or GSPE (final concentration 0, 10, 25, and 50 mg/L) were added into the medium at the same time for 24 h. Each experiment was repeated three times.

### 2.3. Inhibition of Nrf2 Expression

ML385 [20] was used to inhibit the expression of Nrf2. The concentration of ML385 standard was 10 mmol/L. The medium without penicillin-streptomycin was used to dilute the standard to 2, 4, 6, 8, and 10 *μ*mol/L. L-02 cells were treated with the diluted standard for 48 and 72 h. The optimal intervention concentration and intervention time were screened according to Nrf2 expression; see Figure S1.

### 2.4. Detection of Indicators

#### 2.4.1. MTT Viability Assay

MTT (3-(4,5-dimethylthiazol-2-yl)-2,5-diphenyltetrazolium bromide) is a tetrazolium dye that is reduced by NAD(P)H-dependent cellular oxidoreductase enzymes, primarily within the mitochondria of viable cells, to yield an insoluble formazan derivative, which can be solubilized and assayed colorimetrically as an indicator of cell viability. L-02 cell lines were seeded (about 5 × 10^3^ cells were added at 100 *μ*L per well) in 96-well plate. Cells were treated with As or GSPE after adherence at 37°C and 5% CO_2_ atmosphere for 12, 24, and 48 hours. Results were expressed as survival rate, with 100% representing control cells. MTT data were obtained from duplicate wells per treatment shown for three independent experiments.

#### 2.4.2. Annexin V-FITC/Propidium Iodide Apoptosis Assay

The percentage of early apoptosis and necrosis was measured using an annexin V-FITC/propidium iodide (PI) apoptosis kit for flow cytometry, according to the manufacturer's instructions (Invitrogen, Grand Island, NY, USA). After treatment, the cells were harvested, washed twice with phosphate-buffered saline (PBS), and then incubated with 5 *μ*L FITC-annexin V and 1 *μ*L PI working solution (100 *μ*g/mL) for 15 min in the dark at 37°C. Cellular fluorescence was measured by flow cytometry analysis using a flow cytometer (FACSCalibur, BD Biosciences, CA, USA).

#### 2.4.3. Measurement of ROS

2′,7′-Dichlorodihydrofluorescein diacetate (DCFH-DA) fluorescent labeling was used to measure intracellular ROS production in L-02 cells. For the procedure, L-02 cells were exposed to GSPE (10, 25, and 50 mg/L), arsenic (25 mM), or arsenic + GSPE for 24 h. Then, the cell supernatants were removed and DCFH-DA was added to each group. After incubation with DCFH-DA for 30 min at 37°C, the cells were washed twice with PBS and maintained in 1 mL serum-free medium. The fluorescence images were captured by a fluorescence microscope (OLYMPUS U-RFLT50, Japan) under ×100 magnification, with a filter at excitation and emission wavelengths of 500 and 525 nm, respectively.

#### 2.4.4. Detection of Oxidative Stress and Liver Function

GSH specifically deoxidizes dithiobisnitrobenzoic acid (DTNB) to form a yellow product 2-nitro-5-SH-benzoic acid, which can be measured by colorimetry at 532 nm. SOD activity was measured using a tetrazolium salt for detection of superoxide radicals generated by xanthine oxidase and hypoxanthine. One unit of SOD is defined as the amount of enzyme needed to exhibit 50% dismutation of the superoxide radical at 37°C. The reaction product was measured at 450 nm. MDA, a marker of lipid peroxidation, was measured with a commercial kit according to the manufacturer's instructions. Briefly, the samples were treated with thiobarbituric acid, which produces a red compound with an absorption maximum at 532 nm in the presence of MDA. The concentration of MDA was calculated by comparing its absorbance to that produced by the standard, 1,1,3,3-tetraethoxypropane. DTNB can react with compounds containing -SH to form a yellow compound.

At 37°C and pH 7.4, ALT and AST can react with alanine and *α*-ketoglutarate, respectively, to form pyruvic acid and glutamic acid. However, DNPH can terminate the reaction and react with pyruvic acid to form phenylpyruvate, which is rufous under alkaline conditions.

#### 2.4.5. Determination of Arsenic Methylation

High-performance liquid chromatography-hydride generation atomic fluorescence spectra (HPLC-HGAFS) method was used to determine the methylation products of arsenic inside and outside cells, including iAs^3+^, iAs^5+^, MMA, and dimethylarsinic acid (DMA). Cells and culture media were collected after completion of cell intervention. After cell disruption, the cells (200 *μ*L) were filtered with 0.2 *μ*m filtration membrane. Chromatographic eluent was 15 mmol/L (NH_4_)_2_HPO_4_ solution (pH = 6.0, filtered with 0.45 *μ*m fiber membrane before use), and the flow rate was 1.0 mL/min. The negative pressure of the photomultiplier tube was 285 V. The total current of the hollow cathode lamp was 80 mA, and the auxiliary current was 36 mA. The flow rate of carrier gas was 400 mL/min. The current-carrying was 7% hydrochloric acid. The reducing agent included 1.5% KBH_4_ solution and 0.35% KOH mixture. The chromatographic column needs to be calibrated for 30 minutes before use. The percentage of iAs^3+^, iAs^5+^, MMA, and DMA, as well as primary methylation index (PMI) and secondary methylation index (SMI) were calculated.

(1) $$\begin{array}{c} PMI=\frac{DMA}{total\;arsenic\;\left(TAs\right)},\\ SMI=\frac{DMA}{MMA+DMA}. \end{array}$$

In addition, arsenic methylation results were detected at 12, 24, and 48 h. To evaluate the arsenic methylation capacity of cells at each period, we introduced two new concepts: average growth rate of methylation and methylation average speed in the corresponding period. For example, 12 h–24 h average growth rates of monomethylation = (MMA 24 h + DMA 24 h − MMA 12 h − DMA 12 h)/(TAs 24 h − MMA 12 h − DMA 12 h), 12 h–24 h average growth rates of dimethylation = (DMA 24 h − DMA 12 h)/(MMA 24 h + DMA 24 h − DMA 12 h), 12 h–24 h monomethylation average speed = (MMA 24 h − MMA 12 h + DMA 24 h − DMA 12 h)/12 h, and 12 h–24 h dimethylation average speed = (DMA 24 h − DMA 12 h)/12 h.

#### 2.4.6. Detection of mRNA of Nrf2-Related Genes by Real-Time Polymerase Chain Reaction

Total RNA was extracted by TRIzol extraction method (Invitrogen), according to the manufacturer's instructions. Equal amounts of RNA (2 *μ*g) were reverse-transcribed into cDNA using the Transcriptor First-Strand cDNA Synthesis Kit (Roche, Indianapolis, IN, USA). The primers were synthesized by Sigma-Aldrich (St. Louis, MO, USA) for the following genes (Table 1).

All samples were tested in triplicate [3]. Real-time quantitative polymerase chain reaction (qRT-PCR) was performed on a mixture containing 10 *μ*L PCR Supermix (Bio-Rad Laboratories, Hercules, CA, USA), 1 *μ*L forward and reverse primers (Sangon, Beijing, China), 1 *μ*L template DNA, and 8 *μ*L distilled water. The qPCR conditions were as follows: one cycle of initial denaturation (94°C for 3 min), 30 cycles of amplification (94°C for 30 s, 57°C for 30 s, and 72°C for 25 s), one cycle of melting curve measurement (95°C for 5 s, 65°C for 60 s, and a gradual increase in temperature to 97°C), and a cooling period (40°C for 30 s). The data presented were mRNA levels normalized relative to *β*-actin.

#### 2.4.7. Detection of Protein Expression of Nrf2-Related Proteins by Western Blotting

L-02 cells were homogenized in one volume of sample buffer (50 mM Tris-Cl, 100 mM DTT, 10% glycerol, and 2% sodium dodecyl sulfate (SDS)) and centrifuged at 14800 ×*g* at 4°C for 15 min to remove debris. The samples were subjected to SDS-polyacrylamide gel electrophoresis and transferred to polyvinylidene difluoride membranes. After blocking with skim milk (5%), the blots were probed with primary antibodies (Abcam, Cambridge, UK) for Nrf2 (1 : 1000), HO-1 (1 : 1000), NQO1 (1 : 1000), GST (1 : 1000), and *β*-actin (1 : 1000) at 4°C for 8 h. Incubation with primary antibodies was followed by incubation with secondary antibodies (conjugated to horseradish peroxidase) after washing in Tris-buffered saline and Tween 20. The blots were processed using an enhanced chemiluminescence (ECL) kit (Santa Cruz Biotechnology Inc.) and exposed to film. All experiments were repeated three times.

### 2.5. Statistical Analysis

The results were expressed as the mean ± standard deviation. Analysis of variance (ANOVA) was used to detect differences among experimental groups (control, arsenic, GSPE, and arsenic + GSPE). ANOVA was followed by pairwise comparisons with Bonferroni's multiple comparison tests. The data were analyzed using SPSS software for Windows version 17.0 (SPSS Inc., Chicago, IL, USA). A *P* value < 0.05 was considered statistically significant.

## 3. Results

### 3.1. Effects of GSPE and Arsenic on Cell Viability

We first examined the effects of GSPE and arsenic on cell viability by MTT assay. Cell viability decreased significantly with increase in concentration and intervention time of arsenic (*P* < 0.05) when compared with the control group. However, after 12 and 24 h of GSPE intervention, the cell activity did not change significantly (*P* > 0.05) (Figure 1).

To confirm the protective effects of GSPE on arsenic-induced cytotoxicity, cell apoptosis was examined by flow cytometry. GSPE did not induce noticeable apoptosis of L-02 cells (Figure 2(a2, a3, and a4)), while arsenic exposure resulted in significant apoptosis (Figure 2(b1)). All these changes were mitigated by GSPE (Figure 2(b2, b3, and b4)).

### 3.2. GSPE Alleviated Oxidative Stress and Liver Damage Induced by Arsenic

In our study, we found that ROS fluorescence intensity was significantly higher in the arsenic group (Figure 3(e)) than in the control group (Figure 3(a)). However, GSPE effectively removed ROS induced by arsenic (Figures 3(f)–3(h)). Further quantitative detection of ROS in cells was performed by flow cytometry, and similar results were obtained (Figure 4).

We tested the activities of ALT and AST in culture medium and found that ALT and AST activities in the arsenic group were markedly higher than those in the control group (*P* < 0.05). Arsenic + GSPE treatment decreased the activities of ALT and AST compared with the arsenic group (Figure 5).

We used arsenic as an exogenous oxidative stressor in cells. See Figure 6. We tested GSH, SOD, and -SH levels in cells to assess the effects of arsenic on the antioxidant system. Treatment with arsenic caused a prominent decrease in GSH, SOD, and -SH levels compared with the control group (*P* < 0.05). MDA content was significantly higher in the arsenic group than in the control group (*P* < 0.05). As shown in Figure 6, treatment with arsenic + GSPE elevated GSH, -SH, and SOD levels in L-02 cells compared with the arsenic group. In addition, the arsenic + GSPE group had a lower MDA content than the arsenic group. Hence, GSPE reduced oxidative stress induced by arsenic.

### 3.3. Effects of GSPE on Arsenic Methylation

To investigate the effects of GSPE on arsenic methylation, we examined the contents of different valence states of arsenic in L-02 cells, including iAs^3+^, iAs^5+^, MMA, and DMA. Treatment with 50 mg/L GSPE caused a marked decrease in iAs^3+^ levels compared with the arsenic group (*P* < 0.05). However, MMA content was significantly higher in the 25 and 50 mg/L GSPE groups than in the arsenic group (*P* < 0.05). DMA content in each GSPE group was higher than that in the arsenic group (*P* < 0.05; Figure 7).

Furthermore, the proportions of various arsenic compounds in cells and medium were calculated. Compared with the GSPE untreated group, 25 and 50 mg/L GSPE reduced the proportion of iAs3+ (*P* < 0.05) and increased the proportion of iAs5+, MMA, and DMA (*P* < 0.05) in cells. Similarly, treatment with GSPE for 24 h increased the proportion of DMA in medium compared with the untreated group (Figure 8). PMI and SMI were calculated, and the results showed that GSPE significantly increased PMI and SMI in a dose-dependent manner (*P* < 0.05; Table 2).

To explore the effect of GSPE on arsenic methylation further, the average growth rate of methylation and average methylation speed were calculated. We found that the average growth rates of monomethylation and dimethylation in the GSPE treatment groups at 12, 24, and 48 h were higher than those in the GSPE untreated group (*P* < 0.05; Figures 9(a) and 9(b)). Furthermore, GSPE promoted the average methylation speed of monomethylation and dimethylation at 12, 24, and 48 h compared with the GSPE untreated group (Figures 9(c) and 9(d)).

### 3.4. Changes in the Nrf2 Signal Pathway

L-02 cells were treated with arsenic (25 *μ*M) and GSPE (10, 25, and 50 mg/L) for 24 h, and the mRNA and protein expression of Nrf2 and its target genes were detected by qRT-PCR and western blotting. We found that treatment with GSPE (25 and 50 mg/L) significantly elevated the protein contents of Nrf2, NQO1, HO-1, and GST in a dose-dependent manner compared with the control group (*P* < 0.05). Compared with the control group, arsenic (25 *μ*M) markedly decreased the protein expression of Nrf2 and its downstream genes after 24 h (*P* < 0.05). However, the protein contents of Nrf2, NQO1, HO-1, and GST in the arsenic + GSPE group increased gradually compared with the contents in the arsenic group (Figures 10 and 11). Similar trends were observed for mRNA expression of Nrf2 and its downstream genes (Table 3).

### 3.5. Changes in Liver Function and Oxidative Stress after Nrf2 Inhibition

ML385 (5 *μ*M) was used to inhibit the expression of Nrf2. ALT and AST levels in the arsenic group after Nrf2 inhibition were significantly higher than those in the control group (*P* < 0.05) and higher than those in the arsenic group before Nrf2 inhibition (*P* < 0.05). After Nrf2 inhibition, high-dose GSPE could still reduce ALT and AST levels compared with the arsenic group, but the reducing effect of GSPE on arsenic-induced ALT and AST levels was weak (Figure 12).

Oxidative stress indicators were detected after Nrf2 inhibition. We found that 50 mg/L GSPE could increase SOD activity and reduce MDA level compared with the control group (*P* < 0.05). SOD, GSH, and -SH levels in the arsenic group decreased further after Nrf2 inhibition (*P* < 0.05) when compared with the control group and were lower than those in the arsenic group before Nrf2 inhibition (*P* < 0.05). MDA content increased further after Nrf2 inhibition (*P* < 0.05) and was higher than that in the arsenic group before Nrf2 inhibition (*P* < 0.05). SOD and -SH levels in the arsenic + GSPE group increased after Nrf2 inhibition (*P* < 0.05) compared with the levels in the arsenic group, but were still lower than the levels in the arsenic + GSPE group before Nrf2 inhibition (*P* < 0.05; Figure 13).

### 3.6. Role of Nrf2 in Arsenic Methylation

After Nrf2 inhibition, treatment with 50 mg/L GSPE caused a prominent increase in iAs^3+^ levels compared with the same intervention in Nrf2 normal cells (*P* < 0.05). However, DMA content in the 50 mg/L GSPE group after Nrf2 inhibition was lower than that in Nrf2 normal cells treated with the same dose (*P* < 0.05). In Nrf2-suppressed cells, GSPE had no significant effect on MMA compared with Nrf2 normal cells (*P* > 0.05). In addition, MMA content in Nrf2-suppressed cells was higher than that in Nrf2 normal cells (*P* < 0.05) (Figure 14).

Furthermore, the proportions of various arsenic compounds in Nrf2-suppressed cells and its medium were calculated. The iAs^3+^ proportion was higher in Nrf2-suppressed cells treated with GSPE (50 mg/L) than in Nrf2 normal cells treated with the same dose (*P* < 0.05). However, the DMA proportions in Nrf2-suppressed cells treated with GSPE (50 mg/L) and in medium were lower than that in Nrf2 normal cells and medium treated with the same dose (*P* < 0.05) (Figure 15).

Table 4 shows that the SMI was lower in Nrf2-suppressed cells treated with GSPE (50 mg/L) than in Nrf2 normal cells treated with the same dose (*P* < 0.05). The average growth rate of methylation and average methylation speed in Nrf2-suppressed cells were calculated. We found that between 0 and 12 h, the average growth rate of dimethylation in Nrf2-suppressed cells of each group cells was lower than that in Nrf2 normal cells treated with the same doses (*P* < 0.05). Between 12 and 24 h, the average growth rate of monomethylation in each GSPE group and the average growth rate of dimethylation of the GSPE (25 and 50 mg/L) group were lower (*P* < 0.05) in Nrf2-suppressed cells than in Nrf2 normal cells treated with the same doses. Between 24 and 48 h, the average growth rate of monomethylation in each GSPE group and the average growth rate of dimethylation of the GSPE (50 mg/L) group were lower (*P* < 0.05) in Nrf2-suppressed cells than in Nrf2 normal cells treated with the same doses (Figures 16(a) and 16(b)).

We calculated the average methylation speed of monomethylation and dimethylation as well. Between 12 and 24 h, the average methylation speed of monomethylation and dimethylation in Nrf2-suppressed cells treated with GSPE (10 and 50 mg/L) was lower than that in Nrf2 normal cells treated with the same doses (*P* < 0.05). Between 24 and 48 h, the average methylation speed of monomethylation and dimethylation in Nrf2-suppressive cells treated with GSPE (25 and 50 mg/L) was lower than that in Nrf2 normal cells treated with the same doses (*P* < 0.05; Figures 16(c) and 16(d)).

### 3.7. Effects of GSPE on the Nrf2 Pathway after Nrf2 Inhibition

The mRNA expression of Nrf2 and its downstream genes significantly decreased after Nrf2 inhibition. In Nrf2-suppressed cells, low-dose GSPE had no significant effect on the mRNA expression of Nrf2 and its downstream genes (*P* > 0.05) compared with the control group. In Nrf2-suppressed cells, GSPE could still mitigate arsenic-induced decrease in mRNA expression of Nrf2 and downstream genes; however, its effect was weaker than that in Nrf2 normal cells (Figure 17). Similar effect was found in the expression of Nrf2 and its downstream proteins (Figure S2).

## 4. Discussion

In this study, we aimed to determine the effects of GSPE on oxidative damage and arsenic methylation and to clarify the role of Nrf2 in the process. We found that GSPE activates the Nrf2 signaling pathway to antagonize arsenic-induced oxidative damage and to promote arsenic methylation metabolism.

Arsenic exposure can cause liver fibrosis, cirrhosis, and even liver cancer in severe cases [21]. Therefore, analyzing the hepatotoxicity of arsenic and its toxic action mechanism is of great importance for preventing and treating arsenic poisoning. Proanthocyanidins are a type of powerful free radical scavenger and antioxidant found in nature. In this study, arsenic was found to inhibit the Nrf2 signaling pathway, which led to oxidative damage of cells and cell apoptosis. Moreover, the cytotoxic effect of arsenic is closely related to its metabolism in cells. GSPE can activate the Nrf2 signaling pathway and antagonize arsenic-induced oxidative damage, promote arsenic methylation metabolism, and accelerate the metabolism and excretion of arsenic to reduce cell damage. The results of this experiment also provide the basis and evidences for future studies on the action mechanism of arsenic and proanthocyanidins.

Our study showed that arsenic changed the morphology and structure of cells. Arsenic also decreased cell activity and increased apoptosis. Arsenic is cytotoxic and can cause liver damage, and this aspect is speculated to be related to the fact that arsenic can cause oxidative stress in cells [22, 23]. On the other hand, arsenic may inhibit the expression of Bcl2 [24] leading to apoptosis. When proanthocyanidins were treated alone, no significant change in cell activity, apoptosis, and liver function were observed. Therefore, proanthocyanidins have been identified as a safe antioxidant [25]. Moreover, proanthocyanidins could significantly improve cell activity reduction and apoptosis induced by arsenic, indicating that they could antagonize the cytotoxicity of arsenic. These activities are speculated to be related to the antioxidation of proanthocyanidins. Another possibility is that proanthocyanidins promoted the expression of Bcl2 and inhibited apoptosis.

Oxidative stress is one of the action mechanisms of arsenic. Our study proved that arsenic can cause oxidative damage to cells probably via ROS generation [26], antioxidant enzyme reduction [27], and MDA production. In addition, GSH could easily combine with iAs^3+^ and other trivalent arsenides [28], resulting in the reduction of GSH. Moreover, GSH is used during the methylation process of iAs^3+^ [29]. Arsenic can reduce the expression of Nrf2 and its downstream genes. The reduction of antioxidant enzymes induced by arsenic was more obvious in Nrf2-suppressed cells, indicating that arsenic may inhibit the Nrf2 pathway [30, 31] and reduce antioxidant capacity. The mechanism by which arsenic inhibits Nrf2 expression may involve acceleration of Nrf2 degradation by promoting Keap1 protein expression [32]. Proanthocyanidins can improve oxidative damage induced by arsenic [33, 34]. However, the effect of proanthocyanidins on antioxidant enzymes was significantly decreased in Nrf2-suppressed cells. Furthermore, proanthocyanidins could promote the expression of Nrf2 and its downstream genes. It indicated that Nrf2 plays an important role in the action of proanthocyanidins. The underlying mechanism may be through promotion of Nrf2 dissociation from Keap1 [35], after which Nrf2 enters the nucleus to combine with antioxidant responsive element (ARE) on DNA [36], which induces the expression of its downstream antioxidant enzymes. Proanthocyanidins contain a large amount of H^+^, which can block free radical chain reaction, thus improving the activity of various antioxidant enzymes and antioxidant substances in cells. See Figure 18.

Arsenic toxicity is also closely related to its metabolism in cells. Trivalent arsenic compounds, which have a high affinity to sulfhydryl, are more easily absorbed by the cells than any other valence states of arsenic. Therefore, trivalent arsenic can inhibit the activity of enzymes that contain sulfhydryl; consequently, cell respiration, division, and proliferation are affected and cell metabolism is disturbed [37, 38]. Epidemiological studies have reported individual differences in arsenic methylation, and people with weak methylation are more sensitive to arsenic-induced health damage [39]. It has been found that curcumin and sodium mercaptosulfonic acid can promote the metabolism and excretion of arsenic in mouse [40] and Chang liver cells [41], and these effects are considered to be related to the activation of the Nrf2 signaling pathway. In our study, we found that GSPE can promote arsenic methylation metabolism in cells and improve the arsenic methylation ability. After Nrf2 inhibition, the cells still showed methylation metabolism ability, and GSPE improved the arsenic metabolism ability of the cell. However, arsenic methylation ability in Nrf2-suppressed cells was inferior to that in normal cells, and the effect of GSPE on arsenic metabolism in Nrf2-suppressed cells was weaker than that in normal cells. In addition, GSPE significantly improved the dimethylation capacity of arsenic compared with the monomethylation ability. These findings suggest that GSPE can promote arsenic methylation metabolism in L-02 cells, improve the arsenic methylation ability of cells, especially dimethylation metabolism, reduce the action time of MMA to cells, and decrease toxicity of arsenic to cells.

At present, endemic arsenism is still a worldwide public health problem, and our study found that proanthocyanidins have a good effect on the liver damage caused by arsenic. In addition, proanthocyanidins have been widely used in many fields such as medicine, foods, and cosmetics, and the safety of proanthocyanidins has been well verified [42]. Proanthocyanidins have been used in the adjuvant therapy of patients with obstructive sleep apnea hypopnea syndrome (OSAHS) [43]. Therefore, we believe that proanthocyanidins can be used as a potential adjuvant therapy for arsenic poisoning. For example, arsenic poisoning people can eat more fruits rich with proanthocyanidins and take some proanthocyanidins nourishment while receiving treatment. Procyanidins can also be added to people's daily diet in a right amount.

There is a limitation to this study. ML385 was used to inhibit the Nrf2 signaling pathway and reduce the expression of Nrf2 and its downstream genes for exploring the relationship between proanthocyanidins and the Nrf2 signaling pathway. Since ML385 is an inhibitor of Nrf2 and not a knockout agent, a small number of Nrf2 genes were still expressed.

In conclusion, proanthocyanidins can activate the Nrf2 signaling pathway to antagonize arsenic-induced oxidative damage and to promote arsenic methylation metabolism. Proanthocyanidins can reduce arsenic toxicity and promote arsenic elimination. The Nrf2 signaling pathway plays an important role in the antioxidation process of proanthocyanidins and is of great significance for the prevention and treatment of arsenic poisoning.

## Figures and Tables

**Figure 1:** Viability changes of L-02 cells after arsenic or grape seed procyanidin extract treatment (mean and 95% CI). Cell viability was detected by MTT assay. ^&^12 h versus the control group, *P* < 0.05; ^∗^24 h versus the control group, *P* < 0.05; ^#^48 h versus the control group, *P* < 0.05. CI: confidence interval. Cell viability decreased significantly with increase in concentration and intervention time of arsenic. GSPE had no significant effect on cell viability.

**Figure 2:** Effects of arsenic and/or grape seed procyanidin extract on apoptosis. (a1) The control group showed normal levels of L-02 cell apoptosis. The percentage of apoptotic cells was less than 5%. (a2–a4) GSPE (10, 25, and 50 mg/L for 24 h) treatment groups showed normal L-02 cell apoptosis compared with the control group. In the arsenic (25 *μ*M for 24 h) treatment group, apoptosis increased significantly and was mainly advanced apoptosis (20.2%). (b2–b4) The arsenic (25 *μ*M) + GSPE (10, 25, and 50 mg/L) group (for 24 h) showed gradual decrease in apoptosis with increase in GSPE concentrations.

**Figure 3:** ROS fluorescence intensity in L-02 cells. (a) The control group showed weak ROS fluorescence intensity. (b–d) The GSPE (10, 25, and 50 mg/L for 24 h) groups showed weaker fluorescence intensity than the control group. (e) Intense green fluorescence of ROS was found in the arsenic (25 *μ*M) treatment group. (f–h) The arsenic (25 *μ*M) + GSPE (10, 25, and 50 mg/L) group (for 24 h) displayed gradual decrease in fluorescence intensity with increase in GSPE concentrations. ROS fluorescence intensity was significantly higher in the arsenic group (Figure 3(e)) than in the control group (Figure 3(a)). However, GSPE effectively removed ROS induced by arsenic (Figures 3(f)–3(h)).

**Figure 4:** ROS changes in L-02 cells after arsenic and/or grape seed procyanidin extract treatment for 24 h. The more the number of FITC-A^+^ cells, the more the ROS in the cells: (a1) the control group, (a2) the 10 mg/L GSPE group, (b1) the 25 mg/L GSPE group, (b2) the 50 mg/L GSPE group, (c1) the arsenic (25 *μ*M) group, (c2) the arsenic (25 *μ*M) + 10 mg/L GSPE group, (d1) the arsenic (25 *μ*M) + 25 mg/L GSPE group, and (d2) the arsenic (25 *μ*M) + 50 mg/L GSPE group.

**Figure 5:** Effects of arsenic and/or grape seed procyanidin extract on liver function after 24 h (mean ± SD, *n* = 3). ^∗^Versus the control group, *P* < 0.05; ^#^versus the arsenic group, *P* < 0.05. ALT and AST activities in the arsenic group were markedly higher than those in the control group. Arsenic + GSPE treatment decreased the activities of ALT and AST compared with the arsenic group.

**Figure 6:** Oxidative stress changes in L-02 cells after arsenic and/or grape seed procyanidin extract treatment for 24 h (mean ± SD, *n* = 3). ^∗^Versus the control group, *P* < 0.05; ^#^versus the arsenic group, *P* < 0.05. Treatment with arsenic caused a prominent decrease in GSH, SOD, and -SH levels compared with the control group. MDA content was significantly higher in the arsenic group than in the control group. Treatment with arsenic + GSPE elevated GSH, -SH, and SOD levels compared with the arsenic group.

**Figure 7:** Effect of grape seed procyanidin extract on arsenic methylation (mean ± SD, *n* = 3). ^∗^Versus the arsenic only group, *P* < 0.05. Treatment with 50 mg/L GSPE caused a marked decrease in iAs^3+^ levels compared with the arsenic group. However, MMA content was significantly higher in the 25 and 50 mg/L GSPE groups than in the arsenic group. DMA content in each GSPE group was higher than that in the arsenic group.

**Figure 8:** Proportion of arsenic methylated metabolites in cells and medium (mean ± SD, *n* = 3). The cells were treated with arsenic (25 *μ*M) and grape seed procyanidin extract (GSPE; 10, 25, and 50 mg/L) for 24 h. ^∗^ *P* < 0.05 compared with the GSPE untreated group. Compared with the GSPE untreated group, 25 and 50 mg/L GSPE reduced the proportion of iAs^3+^ and increased the proportion of iAs^5+^, MMA, and DMA in cells. Similarly, treatment with GSPE for 24 h increased the proportion of DMA in medium compared with the untreated group.

**Figure 9:** Effects of grape seed procyanidin extract on average growth rate of methylation and average methylation speed (mean ± SD, *n* = 3). ^#^Versus 0–12 h groups at the same dose of GSPE, *P* < 0.05. The average growth rates of monomethylation and dimethylation in the GSPE treatment groups at 12, 24, and 48 h were higher than those in the GSPE untreated group (a, b). Furthermore, GSPE promoted the average methylation speed of monomethylation and dimethylation at 12, 24, and 48 h compared with the GSPE untreated group (c, d).

**Figure 10:** Western blot analysis of proteins after treatment with arsenic and/or grape seed procyanidin extract. Nrf2, NQO1, HO-1, and GST protein expression was measured in L-02 cells treated with arsenic and/or grape seed procyanidin extract by western blotting. Treatment with GSPE (25 and 50 mg/L) significantly elevated the protein contents of Nrf2, NQO1, HO-1, and GST in a dose-dependent manner compared with the control group. Compared with the control group, arsenic (25 *μ*M) markedly decreased the protein expression of Nrf2 and its downstream genes after 24 h. However, the protein contents of Nrf2, NQO1, HO-1, and GST in the arsenic + GSPE group increased gradually compared with the contents in the arsenic group.

**Figure 11:** Quantitative protein analysis after treatment with arsenic and/or grape seed procyanidin extract. Nrf2, NQO1, HO-1, and GST protein expression levels were measured. *Y*-axis represents protein expression of test protein relative to *β*-actin. Each bar represents the mean ± SD. Significant differences relative to the control and arsenic groups are indicated as follows: ^∗^Versus the control group, *P* < 0.05; ^#^versus the arsenic group, *P* < 0.05.

**Figure 12:** Effects of arsenic and/or grape seed procyanidin extract on liver function after Nrf2 inhibition. After Nrf2 inhibition, L-02 cells were treated with arsenic and/or grape seed procyanidin extract for 24 h. ^∗^Compared with the control group, *P* < 0.05; ^#^compared with the arsenic group, *P* < 0.05. After Nrf2 inhibition, high-dose GSPE could still reduce ALT and AST levels compared with the arsenic group, but the reducing effect of GSPE on arsenic-induced ALT and AST levels was weak.

**Figure 13:** Effects of arsenic and/or grape seed procyanidin extract on oxidative stress after Nrf2 inhibition. After Nrf2 inhibition, L-02 cells were treated with arsenic and/or grape seed procyanidin extract for 24 h. ^∗^Compared with the control group, *P* < 0.05; ^#^compared with the arsenic group, *P* < 0.05. 50 mg/L GSPE could increase SOD activity and reduce MDA level compared with the control group. SOD, GSH, and -SH levels in the arsenic group decreased further after Nrf2 inhibition when compared with the control group and were lower than those in the arsenic group before Nrf2 inhibition. MDA content increased further after Nrf2 inhibition and was higher than that in the arsenic group before Nrf2 inhibition. SOD and -SH levels in the arsenic + GSPE group increased after Nrf2 inhibition compared with the levels in the arsenic group, but were still lower than the levels in the arsenic + GSPE group before Nrf2 inhibition.

**Figure 14:** Effects of grape seed procyanidin extract on arsenic methylation in Nrf2-suppressed cells (mean ± SD, *n* = 3). Nrf2-suppressed cells were treated with arsenic (25 *μ*M) and grape seed procyanidin extract (GSPE; 0, 10, 25, and 50 mg/L) for 24 h. ^∗^Versus the GSPE (0 mg/L) group, *P* < 0.05. Treatment with 50 mg/L GSPE caused a prominent increase in iAs^3+^ levels compared with the same intervention in Nrf2 normal cells. However, DMA content in the 50 mg/L GSPE group after Nrf2 inhibition was lower than that in Nrf2 normal cells treated with the same dose. In Nrf2-suppressed cells, GSPE had no significant effect on MMA compared with Nrf2 normal cells. In addition, MMA content in Nrf2-suppressed cells was higher than that in Nrf2 normal cells.

**Figure 15:** Proportion of arsenic compounds in Nrf2-suppressed cells (mean ± SD, *n* = 3). Nrf2-suppressed cells were treated with arsenic (25 *μ*M) and grape seed procyanidin extract (GSPE; 0, 10, 25, and 50 mg/L) for 24 h. ^∗^Versus the GSPE (0 mg/L) group, *P* < 0.05; ^#^versus the same intervention group in Nrf2 normal cells, *P* < 0.05. The proportions of various arsenic compounds in Nrf2-suppressed cells and its medium were calculated. The iAs^3+^ proportion was higher in Nrf2-suppressed cells treated with GSPE (50 mg/L) than in Nrf2 normal cells treated with the same dose. However, the DMA proportions in Nrf2-suppressed cells treated with GSPE (50 mg/L) and in medium were lower than that in Nrf2 normal cells and medium treated with the same dose.

**Figure 16:** Effects of grape seed procyanidin extract on average growth rate of methylation and average methylation speed in Nrf2-suppressed cells (mean ± SD, *n* = 3). Nrf2-suppressed cells were treated with arsenic (25 *μ*M) and grape seed procyanidin extract (GSPE; 0, 10, 25, and 50 mg/L) for 24 h. ^#^Versus 0–12 h group, *P* < 0.05; red shapes indicate the level in Nrf2 normal cells versus the same intervention group in Nrf2-suppressed cells, *P* < 0.05.

**Figure 17:** mRNA expression of the Nrf2 pathway in Nrf2-suppressed cells (mean ± SD, *n* = 3). L-02 cells were treated with arsenic and/or grape seed procyanidin extract (GSPE) for 24 h. ^∗^In Nrf2 normal cells versus the control group, *P* < 0.05; ^#^in Nrf2 normal cells versus the arsenic group, *P* < 0.05; ^a^in Nrf2 inhibition cells versus the control group, *P* < 0.05; ^b^in Nrf2 inhibition cells versus the arsenic group, *P* < 0.05. In Nrf2-suppressed cells, GSPE could still mitigate arsenic-induced decrease in mRNA expression of Nrf2 and downstream genes; however, its effect was weaker than that in Nrf2 normal cells.

**Figure 18:** The action mechanism of GSPE on oxidative stress induced by arsenic and methylation of arsenic. Arsenic can cause oxidative injuries by reducing the activity of antioxidative enzymes and increasing the amount of peroxide products. GSPE contains many phenolic hydroxyl groups and release H^+^, which can bind active oxygen radicals and competitively block the reaction chains of free radicals, reducing the consumption of antioxidants and increasing the activity of antioxidant enzymes. In addition, GSPE promotes the dissociation of Nrf2 and Keap1 proteins, allowing Nrf2 to enter the nucleus from the cytoplasm, thus promoting the expression of downstream genes of Nrf2 and increasing the antioxidant capacity. The Nrf2 pathway activation increases the level of GSH, which promotes the methylation of arsenic (arrows: promotion; blunt arrows: inhibition).

**Table 1:** qRT-PCR primer design.

Genes	Size	F	R
Nrf2	155 bp	5′-CCCAGCACATCCAGTCAGAAA-3′	5′-AAACGTAGCCGAAGAAACCTC-3′
HO-1	101 bp	5′-GGCCAGCAACAAAGTGCAAGA-3′	5′-TAAGGACCCATCGGAGAAGCG-3′
NQO1	129 bp	5′-CGCAGACCTTGTGATATTCCAGT-3′	5′-GGTCCTTTGTCATACATGGCAGC-3′
GST	246 bp	5′-AGGACCTTGGATGACTTTCTGA-3′	5′-CACCTTTGGCGTTGCGATCTTTT-3′
*β*-Actin	240 bp	5′-CACGATGGAGGGGCCGGACTCATC-3′	5′-TAAAGACCTCTATGCCAACACAGT-3′

**Table 2:** Effect of grape seed proanthocyanidin extract on primary methylation index and secondary methylation index.

Indices	GSPE (mg/L)			
	0	10	25	50
PMI	2.12 ± 0.25	3.25 ± 0.27^∗^	3.89 ± 0.23^∗^	5.06 ± 0.40^∗^
SMI	32.22 ± 1.10	48.30 ± 0.98^∗^	52.70 ± 0.75^∗^	55.28 ± 0.42^∗^

^∗^ *P* < 0.05 versus the GSPE untreated group.

**Table 3:** mRNA expression of Nrf2 and its downstream genes.

Indices	Control	GSPE (mg/L)			As (*μ*mol/L)	As + GSPE		
		10	25	50	25	10	25	50
Nrf2	1.00 ± 0.00	1.19 ± 0.20	1.34 ± 0.27	1.69 ± 0.35^∗^	0.41 ± 0.02^∗^	0.77 ± 0.04	0.99 ± 0.12^#^	1.04 ± 0.11^#^
HO-1	1.00 ± 0.00	1.36 ± 0.20	2.37 ± 0.36^∗^	2.64 ± 0.28^∗^	0.44 ± 0.10^∗^	0.66 ± 0.27	1.03 ± 0.34^#^	2.17 ± 0.12^∗^^#^
NQO1	1.00 ± 0.00	1.57 ± 0.02^∗^	2.21 ± 0.24^∗^	2.67 ± 0.22^∗^	0.50 ± 0.16^∗^	0.62 ± 0.11	1.00 ± 0.18^#^	1.35 ± 0.07^#^
GST	1.00 ± 0.00	1.24 ± 0.05	1.57 ± 0.10^∗^	1.64 ± 0.12^∗^	0.40 ± 0.16^∗^	0.55 ± 0.08^∗^	1.12 ± 0.07^#^	1.45 ± 0.10^∗^^#^

Note: the results were described as mean ± SD (*n* = 3). ^∗^Significant difference from the control group at *P* < 0.05. ^#^Significant difference from the arsenic group at *P* < 0.05.

**Table 4:** Effects of grape seed proanthocyanidin extract on primary methylation index and secondary methylation index in Nrf2-suppressed cells.

GSPE (mg/L)		Nrf2 normal cells		Nrf2-suppressed cells			
		0	50	0	10	25	50
PMI	Mean	2.12	5.06^∗^	1.80	2.71^∗^	3.45^∗^	4.40^∗^
	SD	0.25	0.40	0.22	0.20	0.28	0.32

SMI	Mean	32.22	55.28^∗^	31.02	47.63^∗^	49.43^∗^	51.63^∗^^#^
	SD	1.10	0.42	0.44	0.88	0.40	0.15

^∗^Versus the GSPE (0 mg/L) group, *P* < 0.05; ^#^versus the same intervention group in Nrf2 normal cells, *P* < 0.05.

## Data Availability

The data used to support the findings of this study are available from the corresponding author upon request.

## Supplementary Materials

Supplementary Materials Figure S1. The inhibition effect of ML385 on Nrf2 ML385 was used to inhibit the expression of Nrf2. The concentration of ML385 standard was 10 mmol/L. The medium without penicillin-streptomycin was used to dilute the standard to 2, 4, 6, 8, and 10 *μ*mol/L. L-02 cells were treated with the diluted standard for 48 and 72 h. The optimal intervention concentration and intervention time were screened according to Nrf2 expression. 6 and 10 *μ*mol/L ML385 significantly inhibited Nrf2 expression after 72 h. However, high concentration of ML385 may cause certain cytotoxicity. Therefore, 6 *μ*mol/L and 72 h were selected as the final intervention concentration and intervention time of ML385. Figure S2. Protein expression of the Nrf2 pathway in Nrf2-suppressed cells. The protein expression of Nrf2 and its downstream genes significantly decreased after Nrf2 inhibition. In Nrf2-suppressed cells, 10 mg/L GSPE had no significant effect on the protein expression of Nrf2, NQO1, and HO-1 compared with the control group. 25 and 50 mg/L GSPE could increase the protein expression of Nrf2 and its downstream genes significantly compared with the control group. Arsenic intervention led to further decrease of Nrf2 and its downstream genes than the control group. GSPE could still mitigate arsenic-induced decrease in protein expression of Nrf2 and downstream genes; however, its effect was weaker than that in Nrf2 normal cells.
